RETRACTED

# Guideline and Implementation of Osteosarcoma Nursing Care for Children and Adolescents

**DOI:** 10.1155/2022/2021162

**Published:** 2022-10-11

**Authors:** Qian Gao, Yuhong Yao, Qi Xu

**Affiliations:** ^1^Nursing Department, Department of Bone Oncology, The Second Affiliated Hospital of Zhejiang University School of Medicine, 310009, China; ^2^Nursing Department, Department of Thoracic Surgery, The Second Affiliated Hospital of Zhejiang University School of Medicine, 310009, China

## Abstract

Clinical trials on pediatric oncology use therapeutic techniques with the overwhelming majority of children's cancer patients obtaining therapy via clinical investigation procedures. Medical treatment is scheduled according to a specific protocol for enrolled patients. These protocols often do not refer to nursing care. Nursing care, on the other hand, must complement the medical care specified in the medical research protocol. Safe treatment administration, assessment of treatment responses, patients' and families' education, and communication with the whole medical team are just a few of the critical nursing tasks that should be properly managed. Nursing care standards have been developed in this study to strike a good balance between the procedure for clinical research and the nursing care connected with it. These recommendations outline the nursing activities and considerations that must be made while caring for pediatric cancer patients who are engaged in a specific clinical investigation procedure. The objective of this study is to outline the procedure through which nursing care guidelines could be developed and evaluated. The goal of this study was to find out the involvement of nurses in the process of health education for osteosarcoma and family patients.

## 1. Introduction

The role of the nurse in the care of osteosarcoma patients is crucial. From the moment the patient and the patient's family are informed about the sickness, the nurse gives support and comfort and also clarifies the information of the medical doctor to them. All elements of medical treatment are handled, and the nursing care provider is typically the first point of contact for patients who call the physician's office seeking information or reporting a problem. The nursing care provider schedules and organizes appointments in accordance with the patient's health and, in certain cases, social requirements to give complete treatment with meticulous attention. This message will offer context for the nurse's role in ensuring the patient's and family's entire care. The most common primary bone cancer in children is osteosarcoma, originating from primitive bone-forming (osteoid generating) mesenchymal cells. It is classified as primary or secondary based on other underline conditions and accounts for roughly 20 percent of all primary bone cancers. Osteosarcoma is quite diverse in its presentation, allowing for classification into various subgroups based on the degree of differentiation, location within the bone, and histological profile. These categories exhibit a range of imaging characteristics, demographic characteristics, and biological behavior. Treatment choices and survivorship have significantly improved in recent years because of the tireless efforts of medical, surgical, and scientific advancements [1–3]. Although over the last few years, the quality of life of people with osteosarcoma has improved significantly, the disease's cause remains unknown. Historically, studies aimed at determining the origins of osteosarcoma have emphasized a variety of elements, including genetics, epidemiology, and the environment [4–6]. The very complicated karyotypes characteristic of osteosarcoma tumor cytology have posed difficulties in fully characterizing recurring chromosomal alterations. Nonetheless, research has discovered many genetic abnormalities in primary osteosarcoma patients [7].

RETRACTED

Numerous advancements have been achieved in the delivery of curative medicines to children and adolescents with cancer during the last decade. The majority of advancements in this field are due to the predominance of clinical trials since the majority of pediatric oncology patients are treated according to medical research procedures. Protocol-directed therapy is used in pediatric oncology to discover the best successful treatment for groups of pediatric oncology patients. Additionally, protocols allow health care practitioners to identify treatment response differences that are associated with individuals' genetic makeup, sex, age, and ethnicity [8]. Prior to the 21^st^-century merging of the pediatric oncology cooperative organizations to establish the Children's Oncology Group (COG), a Children's Cancer Group or Pediatric Oncology Group facility was responsible for around 94 percent of pediatric oncology patients [9, 10]. The COG now has over 100 open trials enrolling roughly 5,000 pediatric oncology patients every year (http://www.childrensoncologygroup.org/). These procedures are thorough blueprints outlining the medical care that will be provided to the kid or teenager during their therapy. Treatments are becoming more complicated, and administration of treatment is becoming more difficult as a result of differences in pharmaceutical preparation, dose, infusion rate, and duration, as well as the use of diverse medications in different procedures [11, 12]. Children oncology nurses have greater responsibility when it comes to arranging patient care in such a way that all scheduled treatment may be administered safely to each patient. Essential nursing care consists of informing the patient and his family about the clinical trial, improving communication between members of the protocol team and the patient and his or her family, administering the medication according to the protocol's specifications, functioning as a patient advocate, and analysing and recording the patient's response to therapy [13–15]. Throughout the trial, these critical nursing tasks need to be well performed in an organized way.

RETRACTED

## 2. Nursing Perspective on the Care for the Pediatric and Adults Suffering from Osteosarcoma

### 2.1. Family-Centered Care

The interaction between the medical staff, the patient, the patient's friends, and family is critical. Our institution has adopted family-centered care as a method to define such interaction. “Family-centred care is a philosophy of health care that influences health care policy, programs, facility design, and daily interactions between patients, families, doctors, and other health care providers.” Family-centered care is built on the premise that the family is the real master in their child's care, as well as the primary source of courage and strength. Dignity and respect are essential values, as are cooperation, involvement, and information sharing [16, 17]. We have the finest potential to operationalize these notions in our day-to-day encounters. We must assist and encourage our patients and their families in becoming specialists in tumor care [18].

### 2.2. Patient Tool Development

When our pediatric patients are diagnosed with osteosarcoma, they embark on an unfamiliar and sometimes dangerous road. Our responsibility as advocates and educators for patients and families cannot be overstated. Developing strategies to assist patients in comprehending their sickness and therapy, as well as organizing and expanding on preliminary information, involves sensitivity, visual information, and imagination [19–21].

### 2.3. Treatment of Symptoms and Prevention

To maintain a high quality of life throughout management, it is critical to avoid and/or reduce illness symptoms and treatment side effects. Pain is the most common and probably utmost distressing symptom. Pain is a symptom that requires attention at several places throughout the continuum of treatment. Vomiting, nausea, lethargy, constipation, and decreased appetite are all common treatment side effects [22].

### 2.4. Pain Caused by a Disease

Pain is typically the most prevalent symptom in individuals with osteosarcoma, and it poses a significant danger to the quality of life unless managed properly. When pain is caused by the formation of a localized tumor, which is usually exacerbated with pathologic fracture and over-the-counter painkillers, for example, ibuprofen and acetaminophen become ineffective. Drugs combining a pain killer and the use of oral opioids are typically the next stage. The most successful method for tumor pain reduction is to start therapy as soon as feasible. A self-report should be included in the first pain assessment (things that alleviate and exacerbate pain, location, time of greatest and least pain, character, and severity—using a rating scale), physiologic measures/diagnostic results, parent input, physical examination, and behavioral observation [23]. Future assessments will frequently be matched to the first baseline exam. Correct continual pain evaluation data is priceless. If the pain disappears rapidly after the initiation of treatment, it is believed to indicate a favorable response to therapy. Persistent or increasing pain during chemotherapy is a cause for concern since it typically implies a failure to respond to therapy; imaging and, subsequently, histology corroborate this. Acute pain can suggest a new involvement, such as a pathologic fracture, which might happen in concomitant trauma, as in the instance of a youngster who has just turned over in bed [24, 25].

RETRACTED

### 2.5. Pain after Surgery

Postoperative pain is somewhat expectable. The pain treatment regimen often includes intravenous (IV) or epidural analgesia. The need to continuously evaluate therapy effectiveness cannot be overstated, since pain is a subjective sensation. Patients will heal far faster if they are not restricted by discomfort [26]. With proper pain management, deep breathing and coughing should become more effective after a thoracotomy. Participation in the rehabilitation program is contingent upon adequate pain treatment for patients experiencing local control operations, containing amputation and limb salvage. Nurses are uniquely qualified to optimize the scheduling of pain medicines in the best interests of the patients [27].

### 2.6. The Pain of a Chronic Illness

Pain caused by progressive illness is a complicated issue that needs collaboration with professionals. Patients and their families have a right to believe we offer the resources necessary to manage their suffering [28–30]. We practice at a time when a plethora of novel modalities may be used for patients with extended illnesses. To improve the quality of life of the patient, radiation combined with radiofrequency ablation, nerve blocks, radiosensitizing chemotherapy, cryoablation, and pain medicines are the most frequently employed methods [30].

RETRACTED

## 3. Methodology Used to Improve Guidelines

In 1999, Nursing Fellowship Program was developed by our hospital's Office of Nursing. Nurses should be better promoted in the institution's study objectives. The first batch of nursing research fellows consisted of ten staff nurses. To encourage nurse participation in the research assignment, we examined our institution's and our Office of Nursing's research missions in depth, exposed nurses to a variety of research programs as well as the study infrastructure at our hospital, focused on the goal and kinds of oncology trials in the clinic, and practiced selected research skills [31, 32]. To better engage nurses in the institution's research objective, nursing care rules were developed to determine the similar nursing elements of a high-volume product or especially complicated curative investigation procedures. The nursing research fellows recognized a requirement for nursing service standards, which was later confirmed by the institution administration. A single procedure was chosen (OS99, which is a unique institutional identification for certain procedures). Nursing research colleagues addressed the primary investigator and presented him with the concept of nursing care recommendations. The formulation of the recommendations started when the principal investigator agreed to give his experience as well as assistance in the creation of guidelines and following the nurse leaders in the relevant environment gave safe time for the fellows to produce the nursing upkeep recommendations [33, 34].

## 4. Nursing Care Guidelines' Concept

The term nursing care guidelines is defined as a self-contained paper developed in conjunction with a curative investigation procedure. The guidelines detail the activities taken in nursing care and the reasons behind those actions necessary for administering the medical treatment as well as educating, monitoring, and supporting the patient throughout the protocol's therapy phases. The recommendations provided nurses with a concise basis of protocol-specific information about direct care. The goals of the recommendations are (1) to boost a medical nurse's belief in himself and capacity to deliver good quality hospital care by explaining why certain nursing care activities are taken, (2) to improve the nurse's comprehension and expertise of the clinical investigation procedure, (3) to improve the nurse's capacity to educate patients and their families about the protocols and clinical testing in general, (4) to reduce the possibility of clinical mistakes, and (5) to improve the nurse's capability to inform patients and their families regarding the process and clinical testing in particular [8, 25].

RETRACTED

## 5. The Guidelines' Content

Nursing upkeep recommendations must be comprehensible. The OS99 recommendations were organized into seven pieces dubbed the “remember box” to accomplish this goal. The seven pieces were general protocol goals, risk assessment, diagnostic imaging, chemotherapeutic treatment plans, rehabilitation services, and surgical nursing care after surgery. While every element serves a distinct function, collectively, they offer nurses the whole breadth of nursing care necessary to deliver to patients registered in the OS99 protocol [35]. Additionally, these facts broaden nurses' expertise and enable them to teach patients and their loved ones more effectively.

The “remember box” serves as a reminder to the nurse about the purpose and limitations of the nursing care standards [35, 36]. This segment reaffirms that this is a technique to assist the nurse, emphasizing the need not to utilize the nursing care standards as to substitute for examining the clinical investigation process.  Section 2 details the procedure's core and secondary goals pertaining to nursing care. Within the procedure, risk assignment classifies patients into strata A (minimal risk) and B (great risk) [35]. The segment on diagnostic imaging includes a list of all screening tests that are necessary during the protocol's therapy and an explanation of why each test is required.

The chemotherapy treatment schema section discusses the administration of chemotherapy. Additionally, the medical and hematological laboratory values are stated in this section that must be obtained before the start of the chemotherapy, the kind of patient monitoring that must be performed prior to and following chemotherapy administration, significant toxicities, and precise links to the methodology for clinical research [37]. Due to the critical nature of surgery and rehabilitation services in the care of a pediatric individual registered in the OS99 method, nursing care guidelines pay special attention to each of these challenges [35, 38, 39].

## 6. Implementation of the Nursing Care Recommendations

The investigation colleagues developed an education strategy to familiarise medical nurses with the idea and contents of the nursing care standards. The coworkers then defined the intended audience and devised procedures for assessing the recommendations' robustness as assessed by staff nurses. Even though staff nurses caring for osteosarcoma patients were the major target audience, other employees of the medical team were educated about the guidelines at educational inservices [40]. The 03 clinical disciplines targeted are as follows: (1) a major portion of OS99 therapy is administered in the outpatient care unit (both the specialized portion of the clinic offering the doctor's office and patient care), (2) the inpatient hematology-oncology unit, and (3) the intensive care unit (ICU) (where the patients will start their rehabilitation after surgery). The teaching event, which was led by nursing research fellows, served as an informal inservice for medical regions that had interacted with osteosarcoma patients. These contents were demonstrated to inservices throughout all shifts in clinical settings. For demonstration in a classroom setting, the fellows delivered instructional assemblies at nursing positions. These were organized to improve presence, despite the fact not many of the nurses in the target areas were able to attend. Attendance varied according to patient population and acuity [41, 42].

RETRACTED

The educational workshop included three primary topics: (1) the aim and objective of developing nursing care standards, (2) the information unique to management plan principles, and (3) the nursing care that is provided to patients who are part of the OS99 procedure [35].

The research fellows underlined the recognized difficulties of protocol-driven treatment, as well as how the recommendations might be used to help the nurse and uncover critical nursing behaviors that are not specified in the protocol manuscript. The emphasis was subsequently directed to specific parts of the OS99 method. Throughout this phase of the teaching session, participants were introduced to and taught the fundamental ideas of the medical research procedure [35, 38].

The nursing research fellows explained to the participants that critical components of the medical research protocol were included in the nursing care recommendations to help nurses better comprehend the OS99 procedure [43], though the colleagues indicated that a significant quantity of medical material was purposely omitted to ensure that nursing care standards were not substituted for the medical study procedure. The next section of schooling focused on particular guidelines. The participants examined each portion of the guidelines. The fellows conducted a posttest on all participants to determine the success of the inservice period in teaching staff nurses about this protocol-specific information. Posttest questions included fill-in-the-blank, similar, and false or true. These queries centered on protocol goals, critical nursing activities, and medication-related adverse events [44]. After introducing the nursing care standards to staff nurses who will most likely look after patients who are part of the OS99 study, the recommendations were finalized and put in a prominent, readily reachable binder in all patient care locations.

RETRACTED

## 7. Conclusions

Family-centered treatment is intended to encourage patients and their families to confront the disease's problems head-on to grow in strength. Our objective is to educate family members of patients about the condition and its cure, while also finding out how to tailor the strategy for their requirements and objectives. Refining a large amount of data into digestible pieces allows the art of nursing to flourish. By preserving as much “normal” as possible via outpatient and home chemotherapy, we can promote normal growth and family life. Management of symptoms is crucial for overall health and usually needs a collaborative approach. Our patients now have access to a greater variety of new drugs, pharmaceutical combinations, and therapy modalities than ever before [45, 46].

## Data Availability

All the data regarding this study is available in the manuscript.
